# Construction of Rheumatoid Arthritis Risk Prediction and Medical Image Applications from Rheumatoid Factor Levels

This article has been retracted.

**DOI:** 10.1155/2022/8617467

**Published:** 2022-10-04

**Authors:** Wenrun Li, Sheng Bi, Yu Liang, Hongyan Zhu

**Affiliations:** Department of Medical Laboratory, The First People's Hospital of Yunnan Province, The Affiliated Hospital of Kunming University of Science and Technology, Kunming, Yunnan, China

## Abstract

**Objective:**

To study the value of rheumatoid factor (RF) levels in the risk assessment of rheumatoid arthritis (RA) and combined hypertension and diabetes mellitus (DM) and construct RA risk prediction and medical image applications from rheumatoid factor levels.

**Methods:**

A total of 249 RA patients who were treated in the First People's Hospital of Yunnan Province, and another 149 non-RA people were selected as the controls. The clinical data and the detection results of serum circulating RF_IgA, RF_IgG, and RF_IgM were collected. The receiver operating curve (ROC) and logistic regression were used to analyze the value of RF levels in the risk assessment of RA and combined hypertension and DM.

**Results:**

After adjusting for age, BMI, smoking, drinking, hypertension, and diabetes, logistic regression analysis showed that RF_IgA positive, RF_IgG positive, and RF_IgM positive were all independent risk factors for RA (*P* < 0.05). The area under the curve (AUC) of circulating RF_IgA, RF_IgG, and RF_IgM levels in predicting RA was 0.79 (95% CI: 0.74-0.83, *P* < 0.001), 0.73 (95% CI: 0.68-0.78, *P* < 0.001), and 0.87 (95% CI: 0.84-0.91, *P* < 0.001), respectively. The AUC for predicting RA was 0.88 (95% CI: 0.85-0.92, *P* < 0.001) when combined detection of circulating RF_IgA, RF_IgG, and RF_IgM levels in peripheral blood. After adjusting for age and sex, logistic regression analysis showed that RF_IgA positive, RF_IgG positive, and RF_IgM positive were not independent risk factors for DM in RA patients (*P* > 0.05).

**Conclusion:**

The levels of serum circulating RF_IgA, RF_IgG, and RF_IgM are valuable indicators for predicting the risk of RA, but not for the risk of RA complicated with hypertension and DM.

## 1. Introduction

Rheumatoid arthritis (RA) is a disease characterized by chronic inflammation of joint synovium, joint destruction, and pannus formation; the incidence of RA worldwide is about 1%, and the incidence of women is 2 to 3 times that of men [1–4]. If RA patients are not properly treated in the early stage, it will adversely affect the patient's health, which may eventually lead to joint deformities and loss of function and seriously affect the patients' emotions, quality of life, and social functions [5, 6]. Although some progress has been made in recent years, the treatment of RA is not completely satisfactory because its pathogenesis has not been fully studied. Studies have shown that early aggressive treatment is very important to improve patient outcomes [7]. Therefore, finding new biological markers for predicting the occurrence of RA is of great significance for preventing and improving the prognosis of RA.

Rheumatoid factor (RF) is an autoantibody that binds to the Fc portion of human IgG [8, 9]. RF is frequently found in patients with RA or other autoimmune diseases, but also in nonrheumatic patients and even healthy subjects [10, 11]. Currently, although RF has been used for the diagnosis of RA, the sensitivity is not satisfactory, accompanied by poor specificity, and the probability of false positive is as high as 5% to 10% [12, 13].

Studies have shown that hypertension is one of the main risk factors for cardiovascular disease in RA patients [14–16], and they may be linked by factors such as inflammatory mediators, immune responses, endothelial dysfunction, and oxidative stress [17]. Studies have found that the incidence of diabetes mellitus (DM) in RA patients is higher than that of the general population, and abnormal glucose metabolism has also been confirmed [18, 19]. Our understanding of the complex mechanisms of RA complicated with hypertension and diabetes is far from enough. In order to reduce the burden of cardiovascular disease in RA patients, obtain the direction of early intervention, reduce the risk of RA complicated by hypertension and diabetes, and improve the health status of patients, we need to conduct advanced research on traditional risk factors.

## 2. Materials and Methods

### 2.1. Subjects

We selected 249 RA patients admitted to the First People's Hospital of Yunnan Province from January 2014 to February 2022 as the research subjects. Inclusion criteria: (1) 18 years and above. (2) The diagnosis of RA was made according to the American College of Rheumatology (ACR) [20]. (3) The clinical data of the subjects were complete and traceable. Exclusion criteria: (1) Combined with other rheumatic diseases such as systemic lupus erythematosus, Sjögren's syndrome, severe knee osteoarthritis, etc. (2) Combined with other rheumatic immune diseases, acute infection, severe liver, and kidney dysfunction (transaminase increased more than 3 times or glomerular filtration rate < 15 ml/min∗1.73m^2^). (3) Suffering from tumors, severe hematopoietic system, and endocrine system diseases. (4) The clinical data of the subjects were incomplete or not traceable. Another 149 healthy subjects were selected as the control group; RA patients were excluded, and they were all over 18 years old with complete clinical data.

### 2.2. Data Collection

The clinical data we collected in this study included subjects' age, sex, body mass index (BMI), smoking history, drinking history, DM history, and hypertension history. Clinical data were derived from patients' diagnosis and treatment data and electronic medical records.

### 2.3. Rheumatoid Factor

In this study, we collected 3 rheumatoid factors, including circulating RF_IgA, RF_IgG, and RF_IgM in peripheral blood. Fasting cubital venous blood was drawn from subjects, and the levels of RF_IgA, RF_IgG, and RF_IgM in peripheral blood were detected by immunoturbidimetry. Positive criteria are as follows: RF_IgA level < 30 IU/mL was positive; RF_IgG level < 20 U/mL was positive, and RF_IgM level < 15 IU/mL was positive.

### 2.4. Statistical Analysis

SPSS (IBM SPSS statistics, version 20.0, SPSS Inc., Chicago, USA) was used for statistical analysis in this study. Continuous variables with normal distribution were expressed as mean ± standard deviation, and a *t*-test was used to compare the differences between the two groups. Continuous variables that did not conform to the normal distribution were expressed as quartiles, and statistical analysis was performed using the independent sample Mann–Whitney *U* test. Enumeration data were expressed by *n* (%), and statistical analysis was performed by *χ*^2^ test. Logistic regression was used to analyze the risk factors of RA after adjusting for age, BMI, smoking, drinking, hypertension, and DM. The receiver operating curve (ROC) was used to analyze the efficacy of circulating RF_IgA, RF_IgG, and RF_IgM levels in predicting RA, and the area under the curve (AUC) and cut-off value were calculated. All assays were two tailed, and *P* < 0.05 indicated a statistically significant difference.

## 3. Results

### 3.1. Clinical Data

The clinical data we collected from RA patients and physically healthy subjects are shown in Table 1. A total of 249 RA patients, the age ranged from 21 to 94 years old, among them, 29.32% were male, and 70.68% were female. The 149 healthy subjects we screened were aged 19-80 years old, of whom 28.86% were male, and 71.14% were female. Results showed that the age and body mass index (BMI) of RA patients were significantly higher than those of the control group, and the proportions of smoking, drinking, DM, and hypertension were also significantly higher than those of the control group, and the differences were statistically significant (*P* < 0.05).

### 3.2. Comparison of RF Levels between RA Patients and Control Groups

The results of the comparison of circulating RF levels in RA patients and controls are shown in Table 2. The results of qualitative analysis showed that the positive rates of RF_IgA, RF_IgG, and RF_IgM in peripheral blood of RA patients were significantly higher than those of the control group, and the differences were statistically significant (*P* < 0.001). Quantitative analysis results showed that the level of RF_IgA in peripheral blood of RA patients was 42.25 (24.56, 81.64) IU/mL; the level of RF_IgG was 24.21 (10.06, 67.33) U/mL, and the level of RF_IgM was 46.32 (7.55, 145.86) IU/mL. The peripheral blood circulating RF_IgA level of the subjects in the control group was 17.96 (7.59, 26.55) IU/mL; the RF_IgG level was 9.40 (5.44, 16.90) U/mL, and the RF_IgM level was 2.78 (1.72, 5.73) IU/mL; the differences were statistically significant (*P* < 0.001). After adjusting for age, BMI, smoking, drinking, hypertension, and DM, logistic regression analysis showed that RF_IgA positive, RF_IgG positive, and RF_IgM positive were all independent risk factors for RA (*P* < 0.05) (Table 3).

### 3.3. Efficacy Analysis of Peripheral Blood Circulating RF Levels in Predicting RA

The ROC was used to analyze the efficacy of circulating RF_IgA, RF_IgG, and RF_IgM levels in predicting RA, and the results are shown in Figure 1. The analysis results showed that the AUC of peripheral blood circulating RF_IgA level in predicting RA was 0.79 (95% CI: 0.74-0.83, *P* < 0.001) (Figure 1(a)); the cut-off value was 28.91 IU/mL, and the sensitivity was 85.91%; the specificity was 63.86%. The AUC of circulating RF_IgG levels in the prediction of RA was 0.73 (95% CI: 0.68-0.78, *P* < 0.001) (Figure 1(b)), with a sensitivity of 83.22% and a specificity of 57.83%. The AUC of peripheral blood circulating RF_IgM level in predicting RA was 0.87 (95% CI: 0.84-0.91, *P* < 0.001) (Figure 1(c)), with a sensitivity of 70.47% and a specificity of 94.38%. The combined detection of circulating RF_IgA, RF_IgG, and RF_IgM levels in peripheral blood predicted RA with an AUC of 0.88 (95% CI: 0.85-0.92, *P* < 0.001) (Figure 1(d)), with a sensitivity of 80.54% and a specificity of 81.45%.

### 3.4. Clinical Data of RA Patients with Hypertension and Nonhypertensive Patients

The comparison results of clinical data of RA patients with hypertension and nonhypertension are shown in Table 4. The results showed that there were no significant differences in age, sex, BMI, smoking, drinking, and DM between RA patients with hypertension and nonhypertensive RA patients (*P* > 0.05).

### 3.5. Comparison of RF Levels in RA Patients with Hypertension and Nonhypertensive Patients

The results of qualitative analysis of RF in RA patients with hypertension and nonhypertensive are shown in Table 5. We found that the proportions of RF_IgA positive, RF_IgG positive, and RF_IgM positive in RA patients complicated with hypertension were not significantly different from those in nonhypertensive RA patients (*P* > 0.05). The levels of RF_IgA, RF_IgG, and RF_IgM in RA combined with hypertension group were [35.36 (20.27, 73.27) IU/mL], [20.54 (9.90, 46.57) U/mL], and [15.57 (7.63, 110.89) IU/mL], respectively. The levels of RF_IgA, RF_IgG, and RF_IgM in nonhypertensive RA patients were [42.65 (25.15, 85.34) IU/mL], [24.56 (69.77, 10.06) U/mL], and [103.30 (7.48, 155.75) IU/mL], respectively. The analysis results showed that the levels of RF_IgA, RF_IgG, and RF_IgM in the RA combined with hypertension group were not significantly different from those in nonhypertensive RA patients (*U* = 1.750, *P* = 0.080; *U* = 1.478, *P* = 0.139; *U* = 1.524, *P* = 0.127).

### 3.6. Clinical Data of RA Complicated with DM and Non-DM Patients

The comparison results of clinical data of RA complicated with DM and non-DM patients are shown in Table 6. The results showed that there were significant differences in age and sex between RA complicated with DM and non-DM RA patients (*P* < 0.05), but there were no significant differences in BMI, smoking, drinking, and hypertension (*P* > 0.05).

### 3.7. Comparison of RF Levels in RA Complicated with DM and Non-DM Patients

The results of qualitative analysis of RF in RA complicated with DM and non-DM patients are shown in Table 7. We found that the proportions of RF_IgA positive and RF_IgG positive between RA complicated with DM patients and non-DM patients were not significantly different (*P* > 0.05). The levels of RF_IgA, RF_IgG, and RF_IgM in RA combined with DM group were [40.55 (20.32, 83.94) IU/mL], [20.21 (8.64, 58.11) U/mL], and [11.40 (7.37, 120.64) IU/mL], respectively. The levels of RF_IgA, RF_IgG, and RF_IgM in non-DM RA patients were [41.25 (24.57, 79.89) IU/mL], [24.56 (10.25, 68.95) U/mL], and [89.48 (7.78, 147.43) IU/mL], respectively. The analysis results showed that the levels of RF_IgA, RF_IgG, and RF_IgM in the RA combined with DM group were not significantly different from those in non-DM RA patients (*U* = 0.213, *P* = 0.832; *U* = 0.696, *P* = 0.487; *U* = 1.164, *P* = 0.245). However, the proportion of RF_IgM positive in RA complicated with DM patients was significantly different from that in RA complicated with non-DM patients (*P* = 0.04) (Table 8).

## 4. Discussion

The results of our study showed that after adjusting for factors such as age, BMI, smoking, drinking, hypertension, and DM, RF_IgA positivity, RF_IgG positivity, and RF_IgM positivity were all independent risk factors for the occurrence of RA. The levels of RF_IgA, RF_IgG, and RF_IgM in peripheral blood were valuable indicators for RA prediction, and the AUCs were all greater than 0.7. The sensitivity of RF_IgA in predicting RA was as high as 85.91%, but the specificity was low, only 63.86%. The sensitivity of RF_IgG to predict RA was as high as 83.22%, but the specificity was low, only 57.83%. The sensitivity of RF_IgM to predict RA was only 70.47%, but the specificity was as high as 94.38%. The combined detection results of RF_IgA, RF_IgG, and RF_IgM had more than 80% sensitivity and specificity in predicting RA. RF_IgA, RF_IgG, and RF_IgM levels were not significantly associated with RA complicated with hypertension and DM.

RA is a systemic autoimmune disease characterized by chronic destructive joint disease. The main clinical manifestations are symmetrical polyarthritis of the hands, wrists, knees, and foot joints, and may also be accompanied by extra-articular manifestations such as fever, anemia, subcutaneous nodules, and major lymph nodes [21, 22]. An epidemiological survey of the Chinese population in 2008 found that the prevalence of RA was 0.2%-0.37%, and there was no significant difference in the prevalence between different regions and ethnic groups [23]. RA has a long course of disease and a high disability rate, which imposes a heavy burden on the patient's family and society. A follow-up study of 8082 RA patients over 5 years found that the annual disability rate of RA patients was as high as 2.5% [24]. If RA patients receive well treatment in the early stage, especially within 3 months of onset, the disease progression will be significantly slowed down, and the disability rate will be significantly reduced [25]. Therefore, early diagnosis and treatment are essential to improve the prognosis of RA patients.

RF is an autoantibody against an epitope on an IgG Fc fragment for the diagnosis of RA. It is one of the RA classification criteria revised by the American College of Rheumatology (ACR) [20]. When RF alone was used as an indicator for diagnosing RA, the specificity is not satisfactory [26, 27], because RF can often be detected in other diseases, such as primary Sjogren's sydrome (PSS), systemic lupus erythematosus (SLE), etc., and the positive rate of RF in healthy people is about 3%-5%; especially in the elderly, the positive rate is about 10%-30% [10, 28]. The results of our study showed that the positive rate of RF_IgA in RA patients was as high as 54.22%; the positive rate of RF_IgG was as high as 50.20%, and the positive rate of RF_IgM was as high as 59.44%; in healthy people, the positive rates of RF_IgA, RF_IgG, and RF_IgM were 12.08%, 8.05%, and 10.74%, respectively. In addition, our research data showed that among subjects aged <60 years old (including RA patients and healthy people), the positive rates of RF_IgA, RF_IgG, and RF_IgM were 33.8%, 32.5%, and 39.6%, respectively. Among subjects aged ≥60 years, the positive rates of RF_IgA, RF_IgG, and RF_IgM were 51.4%, 39.8%, and 45.6%, respectively (data not shown in this study). It suggests that the positive rate of RF increases with age, which is consistent with the results of other studies [29, 30].

We know that the detection of circulating RF_IgA, RF_IgG, and RF_IgM levels has been widely used in the diagnosis of RA with high sensitivity. However, when using a single indicator for diagnosis, there is often a shortage of poor specificity. This conclusion is also confirmed by our study. The AUC sensitivity of RF_IgA and RF_IgG in predicting the occurrence of RA was 85.91% and 83.22%, respectively, but the specificity was only 63.86% and 57.83%. The specificity of RF_IgM in predicting RA was as high as 94.38%, but the sensitivity was only 70.47%. The sensitivity and specificity of the combined prediction of RF_IgA, RF_IgG, and RF_IgM were both above 80%, suggesting that the combined prediction of RF_IgA, RF_IgG, and RF_IgM has greater application value in RA risk assessment.

It is worth noting that the high incidence of cardiovascular disease in RA patients has become a key research topic [17]. Clinical research evidence shows that cardiovascular disease contributes about 40% of the mortality rate of RA patients [31]. A study of 220,000 RA patients from Japan showed that the risk of herpes zoster was significantly increased when RA patients were accompanied by hypertension [32]. In addition, studies have reported that DM is associated with an increased risk of RA [33]. Relevant studies reported that the incidence of RA was 15.1% and 7.6% in patients with DM and without DM, respectively [33]. Another study reported that type 2 diabetes mellitus (T2DM) was associated with an increased risk of RA in women [34]. It can be seen that the occurrence of hypertension and DM in RA patients increases the RA risk. No studies have focused on the role of RF in the risk assessment of hypertension and DM in RA patients. Our study showed that there was no significant difference in the levels of RF_IgA, RF_IgG, and RF_IgM in peripheral blood between hypertensive and nonhypertensive RA patients. RF_IgA positive, RF_IgG positive, and RF_IgM positive were not independent risk factors for RA patients with DM. It suggests that we still have a long way to choose the peripheral blood circulating RF_IgA, RF_IgG, and RF_IgM as the risk assessment indicators for RA complicated with hypertension, and they are not very good choices at present. We estimated the sample size based on the data of the positive rates of RF_IgA, RF_IgG, and RF_IgM in the peripheral blood, and the results showed that the sample sizes required for RA patients and control groups were 18 cases, 11 cases; 17 cases, 10 cases, and 13 cases, 8 cases, respectively. In this study, 249 RA patients and 149 control groups were included, which were significantly higher than the required minimum sample size. Based on our findings, it would be a groundbreaking research to develop a digital application based on medical image applications that can capture potential RA risk after inputting the test results (Figure 2).

However, this study also has some shortcomings. First of all, the clinical anticyclic citrullinated peptide (CCP) also has important significance in the diagnosis of RA. However, in this study, anti-CCP has not been included in the scope of the study, and it cannot be ruled out that the combined detection of anti-CCP and RF can improve the sensitivity and specificity of RA, combined with hypertension and DM risk prediction. Therefore, further related research is needed. In addition, the sample size included in this study is relatively small, and the results of the study with an enlarged sample size are needed to corroborate our conclusions.

## 5. Conclusion

Through our study, it was confirmed that the levels of RF_IgA, RF_IgG, and RF_IgM in peripheral blood are valuable indicators for RA risk prediction, but not for RA combined with hypertension and DM. It is necessary to further supplement the research results of related indicators such as anti-CCP to explore the feasibility of multifactor combined detection to predict the risk of RA, hypertension, and DM.

## Figures and Tables

**Figure 1:** Receiver operating curve (ROC) of circulating RF levels in predicting RA. (a) ROC curve of circulating RF_IgA levels in predicting RA. (b) ROC curve of peripheral blood circulating RF_IgG levels for predicting RA. (c) ROC curve of circulating RF_IgM levels in predicting RA. (d) ROC curve for predicting RA by combined detection of circulating RF_IgA, RF_IgG and RF_IgM levels in peripheral blood. AUC: area under the curve; RA: rheumatoid arthritis; RF: rheumatoid factor.

**Figure 2:** The idea of medical image applications.

**Table 1:** Comparison of clinical data between RA patients and control groups.

Index	RA (*n* = 249)	Control (*n* = 149)	Statistical value	*P* value
Age (years, mean ± SD)	53.32 ± 14.04	47.25 ± 13.02	4.288	<0.001
Sex [*n* (%)]			0.009	0.922
Male	73 (29.32)	43 (28.86)		
Female	176 (70.68)	106 (71.14)		
BMI (kg/m^2^, mean ± SD)	27.54 ± 5.34	26.46 ± 4.85	2.020	0.044
Smoking [*n* (%)]			4.962	0.026
Ever	60 (24.10)	22 (14.77)		
Never	189 (75.90)	127 (85.23)		
Drinking [*n* (%)]			7.009	0.008
Ever	69 (27.71)	24 (16.11)		
Never	180 (72.29)	125 (83.89)		
Hypertension [*n* (%)]			16.777	<0.001
Yes	56 (22.49)	10 (6.71)		
No	193 (77.51)	139 (93.29)		
DM [*n* (%)]			9.781	0.002
Yes	42 (16.87)	9 (6.04)		
No	207 (83.13)	140 (93.96)		

BMI: body mass index; SD: standard deviation; DM: diabetes mellitus; RA: rheumatoid arthritis.

**Table 2:** Comparison of rheumatoid factor levels between RA patients and controls.

Index	RA (*n* = 249)	Control (*n* = 149)	*χ* ^2^ value	*P* value
RF_IgA [*n* (%)]			69.940	<0.001
Positive	135 (54.22)	18 (12.08)		
Negative	114 (45.78)	131 (87.92)		
RF_IgG [*n* (%)]			73.357	<0.001
Positive	125 (50.20)	12 (8.05)		
Negative	124 (49.80)	137 (91.95)		
RF_IgM [*n* (%)]			91.255	<0.001
Positive	148 (59.44)	16 (10.74)		
Negative	101 (40.56)	133 (89.26)		

RA: rheumatoid arthritis;. RF: rheumatoid factor.

**Table 3:** Logistic regression analysis of risk factors for RA.

	B	Std. error	Wald	Df	Sig.	OR (95% CI)
RF_IgA positive	1.072	0.39	7.541	1	0.006	2.920 (1.359-6.274)
RF_IgG positive	1.104	0.423	6.809	1	0.009	3.016 (1.316-6.911)
RF_IgM positive	1.624	0.395	16.875	1	<0.001	5.072 (2.337-11.007)

OR: odds ratio; CI: confidence interval.

**Table 4:** Comparison of clinical data between RA patients with hypertension and nonhypertensive.

Index	Hypertension (*n* = 56)	Nonhypertension (*n* = 193)	Statistical value	*P* value
Age [years, *n* (%)]			0.001	0.976
<60	39 (69.64)	134 (69.43)		
≥60	17 (30.36)	59 (30.57)		
Sex [*n* (%)]			0.019	0.889
Male	16 (28.57)	57 (29.53)		
Female	40 (71.43)	136 (70.47)		
BMI [kg/m^2^, *n* (%)]			2.682	0.102
<25	14 (25.00)	71 (36.79)		
≥25	42 (75.00)	122 (63.21)		
Smoking [*n* (%)]			0.281	0.596
Ever	12 (21.43)	48 (24.87)		
Never	44 (78.57)	145 (75.13)		
Drinking [*n* (%)]			3.502	0.061
Ever	10 (17.86)	59 (30.57)		
Never	46 (82.14)	134 (69.43)		
DM [*n* (%)]			1.072	0.301
Yes	12 (21.43)	30 (15.54)		
No	44 (78.57)	163 (84.46)		

BMI: body mass index; DM: diabetes mellitus.

**Table 5:** Qualitative analysis results of RF_IgA, RF_IgG, and RF_IgM in RA patients with hypertension and nonhypertensive.

Index	Hypertension (*n* = 56)	Nonhypertension (*n* = 193)	*χ* ^2^ value	*P* value
RF_IgA [*n* (%)]			2.668	0.102
Positive	25 (44.64)	110 (56.99)		
Negative	31 (55.36)	83 (43.01)		
RF_IgG [*n* (%)]			1.559	0.212
Positive	24 (42.86)	101 (52.33)		
Negative	32 (57.14)	92 (47.67)		
RF_IgM [*n* (%)]			1.031	0.310
Positive	30 (53.57)	118 (61.14)		
Negative	26 (46.43)	75 (38.86)		

**Table 6:** Comparison of clinical data between RA patients with DM and non-DM.

Index	DM (*n* = 42)	Non-DM (*n* = 207)	Statistical value	*P* value
Age [years, *n* (%)]			27.159	<0.001
<60	15 (35.71)	158 (76.33)		
≥60	27 (64.29)	49 (23.67)		
Sex [*n* (%)]			4.470	0.035
Male	18 (42.86)	55 (26.57)		
Female	24 (57.14)	152 (73.43)		
BMI [kg/m^2^, *n* (%)]			1.709	0.191
<25	18 (42.86)	67 (32.37)		
≥25	24 (57.14)	140 (67.63)		
Smoking [*n* (%)]			0.553	0.457
Ever	12 (28.57)	48 (23.19)		
Never	30 (71.43)	159 (76.81)		
Drinking [*n* (%)]			0.995	0.318
Ever	9 (21.43)	60 (28.99)		
Never	33 (78.57)	147 (71.01)		
Hypertension [*n* (%)]			1.072	0.310
Yes	12 (28.57)	44 (21.26)		
No	30 (71.43)	163 (78.74)		

BMI: body mass index; DM: diabetes mellitus.

**Table 7:** Qualitative analysis results of RF_IgA, RF_IgG, and RF_IgM in RA patients with DM and non-DM.

Index	DM (*n* = 42)	Non-DM (*n* = 207)	*χ* ^2^ value	*P* value
RF_IgA [*n* (%)]			0.362	0.547
Positive	21 (50.00)	114 (55.00)		
Negative	21 (50.00)	93 (45.00)		
RF_IgG [*n* (%)]			0.498	0.481
Positive	19 (45.00)	106 (51.00)		
Negative	23 (55.00)	101 (49.00)		
RF_IgM [*n* (%)]			4.225	0.040
Positive	19 (45.00)	129 (62.00)		
Negative	23 (55.00)	78 (38.00)		

DM: diabetes mellitus.

**Table 8:** Logistic regression analysis of risk factors for RA complicated with DM.

	B	Std. error	Wald	Df	Sig.	OR (95% CI)
RF_IgA positive	-0.238	0.403	0.35	1	0.554	0.788 (0.358-1.736)
RF_IgG positive	-0.147	0.378	0.151	1	0.697	0.863 (0.411-1.812)
RF_IgM positive	-0.553	0.395	1.959	1	0.162	0.575 (0.265-1.248)

OR: odds ratio; CI: confidence interval.

## Data Availability

The data presented in the study are included in the article, further inquiries can be directed to the corresponding authors.
